# Tracheoesophageal Diversion and Laryngotracheal Separation Procedures for Radiotherapy-Related Intractable Aspiration Pneumonia in Nasopharyngeal Carcinoma

**DOI:** 10.1155/2022/2162936

**Published:** 2022-07-23

**Authors:** Wei Gu, Jian Wang

**Affiliations:** ^1^Department of Otolaryngology-Head and Neck, Peking Union Medical College Hospital, Chinese Academy of Medical Sciences and Peking Union Medical College, Beijing, China; ^2^State Key Laboratory of Complex Severe and Rare Diseases, Peking Union Medical College Hospital, Chinese Academy of Medical Sciences and Peking Union Medical College, Beijing, China

## Abstract

**Background:**

Intractable aspiration and aspiration pneumonia are complications after radiotherapy for nasopharyngeal carcinoma (NPC), and they may be life-threatening in severe cases. In the past, the efficacy of controlling aspiration and aspiration pneumonia in such patients was not ideal.

**Objectives:**

We aimed to evaluate the effect of tracheoesophageal diversion and laryngotracheal separation (TED-LTS) procedures for these patients. *Material and Methods*. We retrospectively analyzed the medical data of five patients with intractable aspiration and recurrent aspiration pneumonia caused by NPC radiotherapy who underwent TED-LTS surgery. The patients were evaluated in terms of aspiration pneumonia control, body weight improvement, removal of tube feeding, oral feeding, and complications.

**Results:**

Intractable aspiration and aspiration pneumonia were completely controlled in all cases, and the patients' body weight increased from 46.46 ± 4.6 (38.9-50.3) kg to 55.32 ± 2.7 (51.4-56.7) kg. Four patients were able to consume an oral semisolid diet, and one patient maintained an oral liquid diet. Tube feeding was not required in 4 patients. One patient developed postoperative esophageal fistula, which improved after conservative treatment.

**Conclusion:**

TED-LTS is effective for intractable aspiration and aspiration pneumonia caused by NPC radiotherapy and can be used to restore partial oral feeding. However, strict surgical indications should be followed.

## 1. Introduction

The incidence of nasopharyngeal carcinoma (NPC) is high in South China, Southeast Asia, and among native populations in the Arctic. The number of new cases is 130,000 [1] worldwide. The crude incidence and the mortality rate of NPC in mainland China reported by Wei et al. are much higher than the global levels, at 3.09/100,000 and 1.57/100,000, respectively [2]. The main treatments for NPC are radiotherapy for local lesions [3]. Aspiration is a common and long-term complication after NPC radiotherapy [4]. It is reported that patients with dysphagia symptoms after NPC radiotherapy have an implicit aspiration rate of 42-66% [5–7] with liquid food. The incidence of aspiration pneumonia is also much higher in NPC patients with implicit aspiration than in other populations [8]. It is estimated that the hospitalization rate for aspiration pneumonia after NPC radiotherapy is 3.2%, and the mortality rate of NPC patients within 30 days of hospitalization is 11%-51% [9, 10].

Conventional methods for reducing the occurrence of aspiration pneumonia include oral hygiene, changing the viscosity of food, adjusting the eating position, providing swallowing rehabilitation, and tube feeding. However, due to the existence of gastroesophageal reflux and saliva aspiration, even strict restrictions of ingested food and the use of tube feeding cannot completely prevent life-threatening aspiration pneumonia. For these patients, surgical intervention may be required to protect the airway by preventing the aspiration of saliva, secretions, and reflux contents [11]. Eisele suggested that the ideal surgery for intractable aspiration should be simple, effective, and reversible while preserving both speech and swallowing functions; examples include total laryngectomy, endolaryngeal stents, laryngeal closure, laryngotracheal separation (LTS), tracheoesophageal diversion, and laryngotracheal separation (TED-LTS) [12]. For intractable aspiration, TED-LTS surgery can not only reduce the morbidity and mortality of aspiration pneumonia but can also restore oral or partial oral feeding without the need for tube feeding. It is a recommended surgical method. TED-LTS was first reported in 1975 by Lindeman et al. [13]. The effective rate for the treatment of intractable aspiration was 100%. In these reports, patients who underwent the procedure were mainly those with intractable aspiration caused by neurological diseases. However, TED-LTS is rarely reported for patients with intractable aspiration caused by NPC treatment [14, 15].

This article retrospectively summarizes the data of five patients with recurrent aspiration pneumonia caused by intractable aspiration after radiotherapy who underwent TED-LTS and evaluates its clinical effects.

## 2. Methods

### 2.1. Patients

This study was approved by the Ethics Committee of our hospital, and all patients signed the informed consent form. We conducted a retrospective analysis of the clinical data of five NPC patients who developed intractable aspiration pneumonia after radiotherapy from January 2010 to December 2019. All patients had cranial nerve paralysis, and they suffered from serious vocal cord movement disorders and pharyngeal sensory disorders. Vocal cord movement disorders and pharyngeal sensory disorders were determined by fibrolaryngoscopy. The inclusion criteria were as follows: (1) age younger than 70 years; (2) diagnosis of implicit aspiration and repeated aspiration pneumonia (more than five times) confirmed before surgery; (3) loss of speech function and communicative speech; (4) no response to conservative treatments, such as tube feeding, swallowing rehabilitation, and acupuncture; and (5) no tumor recurrence or distant metastasis. The exclusion criteria were as follows: (1) history of lower neck (level IV, VB) radiotherapy, (2) severe cardiopulmonary dysfunction; and (3) no history of conservative treatment, such as tube feeding.

### 2.2. Surgical Procedure

A transverse incision was made at the anterior lower neck to fully expose the trachea. The trachea was divided between the 4th and 5th rings. The lower end of the divided trachea was anastomosed with the skin, i.e., a tracheostomy was performed. The cartilage of the 4th tracheal ring was removed, preserving the mucosa. The full-thickness esophagus was incised transversely at the level of the 3^rd^ tracheal ring. Then, the upper end of the divided trachea was anastomosed with the esophagus incision in a tension-free manner to form a diverted channel (Figure 1).

### 2.3. Statistical Methods

SPSS v17.0 statistical software (SPSS, Chicago, IL) was used for the descriptive statistical analysis of all data, and quantitative data are expressed as mean ± standard deviation.

## 3. Results

The age of the five patients was 54.8 ± 4.5 (50-61) years with median age as 53. The primary tumor radiotherapy dose was 70.96 ± 1.1 (69.8-72.4) Gy, and no lower neck (level IV, VB) radiotherapy. The time since radiotherapy was 144.4 ± 22.3 (115-176) months. The time since the onset of aspiration pneumonia was 50.8 ± 13.7 (34-70) months. The duration of tube feeding was 26.6 ± 11.1 (12-43) months. The follow-up period was 38.4 ± 15.8 (16-58) months. As of the last follow-up, all patients had survived (Table 1).

Aspiration pneumonia was completely controlled in all patients (Figure 2). The number of occurrences of aspiration pneumonia before the operation was 11.2 ± 3.1 (8-16), and no aspiration pneumonia occurred in the five patients after the operation. Four patients' feeding tubes were successfully removed. Four patients were able to consume a semi-solid diet, and one patient was able to consume a liquid diet. The body weights of the patients were significantly increased from a preoperative body weight of 46.46 ± 4.6 (38.9-50.3) kg to a postoperative body weight of 55.32 ± 2.7 (51.4-56.7) kg (Table 2).

In case 4, esophageal fistula was reported as a postoperative complication. After dressing changes and antibiotic treatment, the wound healed, and the patient was discharged at 24 days after surgery. The remaining patients had no obvious complications.

## 4. Discussion

China is a region with a high incidence of NPC, with nearly 40,000 new cases each year. Radiotherapy is the main treatment for NPC [2]. The high dose of radiotherapy can result in obvious fibrosis of the soft tissue of the head and neck and damage to the posterior cranial nerves located in the radiation field. Nerve damage will also seriously affect sensory and motor function in the patient's throat. Therefore, difficulty swallowing and coughing after NPC radiotherapy are very common complications [14–16]. Although incurable aspiration caused by NPC radiotherapy is rare, it may lead to serious consequences such as aspiration pneumonia, severe malnutrition, and even death if ignored [14, 15].

The nonsurgical methods reported in the literature for reducing aspiration after radiotherapy for NPC include improving oral hygiene, changing the viscosity of food, adjusting the feeding position, providing swallowing rehabilitation, dilating the cricopharyngeal muscle, and tube feeding [11, 17, 18]. Unfortunately, these treatments do not provide satisfactory results for patients with intractable aspiration. Long-term tube feeding and tracheotomy are usually required, but even these interventions cannot completely prevent the occurrence of aspiration pneumonia [11, 19]. Therefore, TED-LTS is the only option for patients with recurrent aspiration pneumonia and life-threatening conditions.

Lei et al. reported nine patients who underwent simple laryngotracheal separation surgery, which completely prevented the occurrence of aspiration pneumonia. However, two patients were unable to be weaned of nutritional support via tube feeding [20]. Our original intention for performing TED-LTS was to restore the patient's oral feeding function by eliminating aspiration pneumonia. The final result was satisfactory. The procedure not only completely resolved the intractable aspiration and aspiration pneumonia but also allowed 4/5 patients to be weaned off the feeding tube. In typical cases, patients with intractable aspiration after NPC radiotherapy also have severe swallowing dysfunction. Simple laryngotracheal separation cannot reconstruct the food passage; in contrast, TED-LTS surgery uses the larynx and trachea as the new “food passage” to improve patients' swallowing function. Moreover, due to the injury of the posterior cranial nerve caused by radiotherapy, these patients have serious implicit aspiration; even if food passes through the larynx and trachea, no cough reflex is triggered. Although the TED-LTS procedure has been performed for many years, very little information is available regarding its utilization after NPC radiotherapy [14, 15]. One of the main reasons for this is that radiotherapy may seriously affect the healing of the anastomosis and cause serious complications. Therefore, we selected patients who did not undergo radiotherapy at the anastomosis site. Because these patients were all at stage N0 and the lower neck was not selected as the radiation area during the first radiotherapy course, the chance of esophageal fistula was minimized. The results show that only one patient had short-term anastomotic fistula. In addition, the removal of the 4th cartilage ring during the operation can achieve a tension-free suture between the trachea and the esophagus. This may be the reason for the reduced occurrence of esophageal fistula. This type of surgery is not only theoretically reversible, but the resulting trauma is relatively small. This presents an advantage over total laryngectomy.

Indeed, although TED-LTS surgery can eliminate the life-threatening condition of recurrent aspiration pneumonia and improve patient quality of life to a certain extent, speech function is sacrificed. Therefore, it is necessary to be cautious when choosing this type of surgery for patients who still have speech function. All the patients in this study had lost their ability to speak before surgery and did not respond to other treatments for life-threatening intractable aspiration and aspiration pneumonia. It should be noted that due to the high-dose radiotherapy in the operation area, there was a certain incidence of esophageal fistula and local infection, so that only 5 patients who had been strictly screened in this study had received the surgery within 9 years. Therefore, the limited sample size is one of the limitations of this study. Other limitations include that this study is a retrospective case series with the lack of the control group, and we focused on limited indicators of concern (only improvement of aspiration pneumonia and oral feeding). In the future study, prospective controlled trials with larger cohorts are needed.

## 5. Conclusion

TED-LTS is effective for the treatment of intractable aspiration and aspiration pneumonia caused by NPC radiotherapy, and it can restore partial oral feeding. However, strict surgical indications should be met.

## Figures and Tables

**Figure 1:** Surgical procedures of the tracheoesophageal diversion and laryngotracheal separation. (a) Schematic diagram of surgical procedure (sagittal position); black arrow indicates the trachea fistula. (b) Schematic diagram of surgical procedure (coronal position), the trachea is divided between the 4th and 5th tracheal rings, the upper end of the divided trachea is anastomosed to the anterior wall of the esophagus, and the lower end is sutured with the skin to create a stoma; black arrow indicates tracheoesophageal anastomosis. (c) Representative intraoperative picture of surgical area after tracheal separation; black arrow indicates the upper end of the divided tracheal and white arrow indicates the anterior wall of esophagus. (d) Representative intraoperative picture of the tension-free anastomosis between the upper end of the divided trachea and the anterior wall of the esophagus; black arrow indicates the thyroid cartilage, and white arrow indicates the tracheoesophageal anastomosis. TC: thyroid cartilage; UT: upper trachea; E: esophagus; LT: lower trachea).

**Figure 2:** The complete control of aspiration pneumonia in one patient. (a) The patient was receiving jejunal tube feeding due to recurrent aspiration pneumonia in 2017. (b) Aspiration pneumonia still occurred one year after tube feeding began. (c) The lung condition had completely improved one year after surgery. (d) A postoperative angiography image taken during swallowing that shows the contrast agent entered the esophagus through the larynx and the tracheal-esophageal anastomosis (blue arrow). (e) At three months after surgery, the fiber laryngoscope passed through the larynx and the trachea. Unobstructed tracheal-esophageal anastomosis was observed, with mild edema in the surrounding areas. (f) Esophageal secretions observed through the anastomotic site.

**Table 1:** Demographic information of five patients enrolled in this study.

Number	Age	Gender	Staging	PSD (Gy)	TR (months)	TP (months)	TFMT (months)	OCTM	TT (months)	DFAS (months)
1	52	Male	T2N0M0	71.8	176	70	Intestine (43)	Rehabilitation, acupuncture	No	58
2	58	Male	T1N0M0	70.2	153	48	Stomach (26)	rehabilitation	Yes (30)	46
3	61	Female	T1N0M0	69.8	140	34	Intestine (12)	rehabilitation	No	40
4	50	Male	T2N0M0	72.4	138	58	Intestine (28)	Rehabilitation, acupuncture	No	32
5	53	Male	T1N0M0	70.6	115	44	Stomach (24)	Rehabilitation	Yes (21)	16

PSD: primary radiotherapy sites and dose; TR: time since radiotherapy; TP: time since the onset of pneumonia; TFMT: tube feeding method and time; OCTM: other conservative treatment methods; TT: tracheotomy and time; DFAS: duration of follow-up after surgery.

**Table 2:** Complications and outcomes of tracheoesophageal diversion and laryngotracheal separation in five patients.

Number	PEF	FRT	BW (kg)		NAPE		Type of diet
			Preoperation	Postoperation	Preoperation	Postoperation	
1	No	Yes	45.6	51.4	16	0	Semisolid diet
2	No	Yes	47.8	55.6	9	0	Semisolid diet
3	No	Yes	50.3	56.7	12	0	Semisolid diet
4	Yes	No	38.9	54.3	8	0	Semisolid diet
5	No	Yes	49.7	58.6	11	0	Liquid diet

PEF: postoperative esophageal fistula; FTR: feeding tube removal; BW: body weight; NAPE: number of aspiration pneumonia events.

## Data Availability

All data needed to evaluate the conclusions in the paper are presented in the paper. Additional data related to this paper can be requested from the authors.
